# Dual role of *KRT17*: development of papillary renal cell tumor and progression of conventional renal cell carcinoma

**DOI:** 10.7150/jca.32579

**Published:** 2019-08-28

**Authors:** Donat Peter Sarlos, Maria V Yusenko, Lehel Peterfi, Arpad Szanto, Gyula Kovacs

**Affiliations:** 1 Department of Urology, Medical School, University of Pecs, Hungary; 2 Institute of Biochemistry, University of Muenster, Germany; 3 Medical Faculty, Ruprecht-Karls-University, Heidelberg, Germany

**Keywords:** KRT17 expression, Kidney cancer, Tumor development, Tumor progression.

## Abstract

Expression of* KRT17* has been described in multi-layered epithelia as well as in tumors derived from these cells. In cancers arising from *KRT17* negative single layered epithelia neo-expression of *KRT17* has been associated with tumor progression. To obtain more insight into the biology of kidney cancers we have investigated *KRT17* expression by immunohistochemistry in normal kidney, in papillary preneoplastic lesions and in 151 papillary and 692 conventional renal cell carcinomas placed on tissue microarray. We found a positive staining in ureteric bud and collecting duct cells in foetal kidney, in all papillary preneoplastic lesions and also in 77% of the 151 papillary renal cell tumors indicating a continuos *KRT17* expression during tumor development. The neo-expression of *KRT17* in conventional renal cell carcinomas, which derives from *KRT17* negative proximal tubules showed a significant correlation with postoperative tumor relapse (RR=2.50; 95% CI=1.59-3.94; p<0.001). In conclusion, the continuous expression of *KRT17* from emerging fetal kidney tubules and microscopic pre-neoplastic lesions towards papillary renal cell tumors and its neo-expression in aggressive growing conventional renal cell carcinomas reflects the multiple function of *KRT17* in kidney cancers with distinct natural history. This should be taken into account in clinical managements and therapy.

## Introduction

Keratins are intermediate filaments playing a crucial role in the integrity and mechanical stability of single epithelial cells and epithelial tissues. The expression of keratins is regulated in a tissue-type and differentiation-specific manner 1. Highly specialized parenchymal epithelial cells, such as tubular cells of the kidney, express only *KRT8* and *KRT18* in their normal state, but this may change during inflammation, regeneration and also during tumor development. Kidney tubular cells may switch on *KRT7* and *KRT19*, sometimes also *KRT17* in addition to the expression of *KRT8* and *KRT18* 1. The increased expression of *KRT7*, *KRT17* and *KRT19* appears parallel to the reduction in degree of differentiation. *KRT7* and *KRT19* are upregulated during renal epithelial injury and repair leading to more plasticity of cells involved in the regeneration processes 2. It was also shown that shift of *KRT8* and *KRT18* expression to *KRT7* and *KRT19* is associated with structural remodelling of end stage kidney and increased frequency of tumors expressing both *KRT7* and *KRT19* 3. The KRT7 is expressed in papillary renal cell tumors (RCT) and also used in the differential diagnosis of renal oncocytoma (RO) and chromophobe renal cell carcinoma (RCC) 4,5. However, the possible involvement of *KRT17* in the biology of kidney cancer is not yet known. Two earlier studies on the keratin expression in distinct types of renal cell cancer using the E3 clone from DAKO did not find *KRT17* expression in conventional, chromophobe and papillary renal cell tumors or renal oncocytoma 4,5.

*KRT17* a member of type I acidic epithelial keratin family was first identified in skin basal cell epithelioma and it is considered to be a basal/myoepithelial cell keratin 6. Expression of *KRT17* occurs in complex, multilayered epithelia and it is largely retained during neoplastic transformation leading to several types of cancer derived from such epithelial cells 7-10. In the last few years *KRT17* expression has also been detected in several tumors of non-epithelial type but not in their tissue of origin. These studies demonstrated a correlation between neo-expression of the *KRT17* and tumor progression 11-16. These findings suggest distinct roles of *KRT17* in fetal development, regeneration and tumorigenesis and on the other hand in the progression of frankly malignant cancers.

In attempt to learn about the involvement of *KRT17* in the biology of renal tumors we applied immunohistochemistry to a large panel of conventional RCC and papillary RCT as well as to preneoplastic lesions (PNL) associated with papillary RCT. In our study we used an antibody arised against the N-terminal protein fragment of *KRT17* instead of the E3 clone from DAKO (Glostrup, Denmark).

## Materials and Methods

### Patients and tissue samples

We have enrolled tumor samples from consecutively operated patients without selection, who undervent radical or partial nephrectomy due to kidney cancer between 2000 and 2013 at the Department of Urology, Medical School, University of Pecs, Hungary. The only criteria was the availability of clinical data, follow-up and paraffin embedded tumor material. Data on regular follow-up and tumor-specific death were obtained from the Registry of the Department of Urology. Follow-up was defined as time from operation until the last recorded control in 2018, or cancer-specific death. Patients who died from causes other than RCC were excluded from this analysis. Preoperative clinical staging included abdominal and chest computed tomography (CT) scans. Bone scans and brain CT scans were obtained only when clinically indicated. The presence of nodal metastases was confirmed by histological, whereas that of distant metastases by radiographic examination. During the postoperative period patients were surveyed every 6 months by abdominal ultrasound scans, serum creatinine and eGFR measurements, and every year by CT scans. Histological diagnoses were performed by a genitourinary pathologist (GK) according to the Heidelberg and TNM classification systems 17,18. Paraffin embedded material from foetal and adult kidneys were obtained from the archive of the Institute of Pathology, Medical School, University of Pecs, Hungary. We have also analysed 17 PNL associated with papillary RCT. All procedures performed in this study were in accordance with the ethical standards of the institutional research committee and with the 1964 Helsinki declaration and its later amendments. The collection and use of all tissue samples for this study were approved by the Ethics Committee of the University Pecs, Hungary (No. 5343/2014).

### Tissue microarray (TMA) and immunohistochemistry

Haematoxylin and eosin stained slides were reviewed to select the representative paraffin blocks and tumor areas for TMA construction. From each tumor minimum three core biopsies with a diameter of 0.6 mm were placed in the recipient block using a Manual Tissue Arrayer (MTA1, Beecher Instruments, Inc., Sun Prairie, CA, USA). For marking the TMAs fetal and adult kidney biopsies were included.

Paraffin blocks of fetal and adult kidneys, pre-neoplastic lesions and TMAs were used for immunohistochemistry. After deparaffinisation and rehydration the 4 um thick sections were subjected to heat-induced epitope retrieval in citrate buffer, pH 6.0 in 2100-Retriever (Pick-Cell Laboratories, Amsterdam, The Netherlands). Endogenous peroxidase activity and unspecific binding sites were blocked with 3% hydrogen peroxide containing 1% normal horse serum for 15 minutes at room temperature. Slides were incubated overnight at 4^0^C in a moist chamber with rabbit polyclonal anti-KRT17 antibody (HPA 000452, lot Nr. A08686, Sigma Aldrich, Budapest, Hungary) at 1:500 dilution. Horse-radish-peroxydase conjugated anti-rabbit, anti-mouse secondary antibody (HISTOLSMR, Histopathology Ltd, Pecs, Hungary) was applied for 30 minutes at room temperature and the bound antibody was visualized with AEC (Amino-ethyl-carbazol) (DAKO, Glostrup, Denmark). Tissue sections were counterstained with Mayer's haematoxylin. In negative control the primary antibody was omitted. The slides were evaluated twice at different times by two of the authors (DPS, GK). The staining intensities were scored as low, medium or high. As we did not find substantial differences between weak or strong *KRT17* expression and conventional RCC progression, we have evaluated all staining intensity as positive.

### Statistical analysis

Data analyses were performed using a SPSS Statistics software package version 25 (IBM, 35 Armonk, NY, USA). Correlations between *KRT17* expression, clinical and pathological parameters were calculated using the χ^2^ test. The effects of the different variables (age, sex, size of tumor, TNM classification, grades, stages, metastases and KRT17 expression) on the survival of the patients were estimated by Kaplan-Meier analyses. Comparisons of survival curves were made using the Log rank test. Univariate and multivariate survival analyses were performed using the Cox regression model. Patients that were alive and disease-free were censored. Differences were considered significant at* p* < 0.05.

## Results

### Expression of *KRT17* in normal fetal and adult kidney

The expression of *KRT17* first appeared in the ureteric bud and collecting duct of fetal kidney (Figure 1A). There was a weak staining of *KRT17* at the tip of the ureteric bud connected to the distal part of the S-shaped body and the staining is intensified along the medullary collecting duct towards the kidney papilla (Figure 1B). In fetal kidney each cell of the collecting duct displayed a positive immunoreaction, no cell type specific selective staining was seen along the tubules. In adult kidney the vast majority but not all cells of the connecting tubules and cortical collecting ducts displayed a strong *KRT17* staining (Figure 1C). The medullary collecting ducts showed a similar selective staining in the vast majority of cells (Figure 1D). In contrast to the fetal kidney *KRT17* expression is restricted to one specific type of epithelial cell in connecting tubules, cortical and medullary collecting ducts of adult kidney. No *KRT17* staining was seen in proximal and distal tubules and loop of Henle.

### Expression of *KRT17* in papillary RCT and associated PNL

We have analyzed the *KRT17* expression in PNL associated with papillary RCT including 8 lesions from two patients with germ line *MET* mutation 17. The protein encoded by *KRT17* was detected in each of the 17 small solid, tubular papillary lesions with 1 to 3 mm in diameter (Figure 1E,F). A diffuse cytoplasmic staining with increased signal attenuated to the cell membrane was seen in 116 of the 151 papillary RCTs (Figure 1G-I). Altogether, we found *KRT17* positivity in 77% papillary RCTs irrespectively of the size of tumor cells such as small, medium or large cell which are considered by others as type I and type II or mixed type.

### Expression of *KRT17* in conventional RCCs is associated with tumor progression

To estimate the role of *KRT17* in postoperative tumor relapse, we set up a Cohort of 692 patients without metastatic tumor at the time of operation. The mean age of the entire cohort was 61.1±11.4 years (range 20-88 years), the average follow-up was 60.6±33.2 months. Out of the 692 patients 108 (16%) developed metastasis during the follow-up and died due to metastatic cancer. The clinical parameters and correlation with* KRT17* expression is shown in Table 1. In this Cohort 94 tumors (14%) displayed positive *KRT17* staining which showed a significant correlation with cancer specific death, tumor size, T-stadium, grade and stage. The Kaplan-Meier analysis indicated that patients with *KRT17* positive tumor have a significantly shorter survival than those with negative tumor (Figure 3). The 5-year cancer specific survival rate for the *KRT17* positive and negative group was 65.2% and 91.5%, whereas the 10-year survival rate was 36.4% and 78.3%, respectively. The multivariate analysis showed a significant correlation between the risk for postoperative tumor recurrence, tumor grade as well as *KRT17* positivity (each <0.001). The *KRT17* expression was an independent negative survival factor indicating a nearly three times higher risk of disease relapse and cancer specific death (RR=2.50; 95% CI=1.59-3.94; p<0.001).

## Discussion

Beyond its role to maintain cellular integrity of multi-layered epithelia *KRT17* has other functions as well. *KRT17* plays a role in fetal epidermal development and in cell proliferation during wound healing by regulation of protein synthesis through intracellular signaling pathways 6, 20. *KRT17* knockout mouse embryos show a delay in closure of surface ectoderm wounds 21. *KRT17* binds and sequester TRADD (TNFRSF1A associated via death domain), a mediator of programmed cell death signaling and protects the cells from apoptosis 22. It was also shown that *KRT17* null keratinocytes are sensitive to TNF mediated apoptosis 22. The onset of *KRT17* expression in embryonic ectoderm reflects its commitment towards distinct epithelial lineages and that the program of gene expression characteristic of wound-activated adult keratinocyte may have a relationship to that executed by epithelial cells at specific stages of embryonic development 23. *CD44*+/*KRT17*+ cells have stemlike properties, including the capacity for cell renewal and in vivo tumorigenicity 24. This finding may explain the role of KRT17 in the maintenance and persistance of embryonal structures, e.g. PNL in differentiated kidneys.

We showed in this study that *KRT17* is expressed in simple (one-layered) epithelial cells of fetal and adult kidney. Each PNL of embryonal origin as well as 77% of papillary RCT showed the *KRT17* positivity irrespectively of cell type. Taking into account that only 5% of papillary RCTs developed metastasis during 5-year follow-up (data not shown), the role of *KRT17* in the progression of papillary RCT can be excluded. Rather, the expression of *KRT17* in fetal kidney suggests that it may play a role in the cell specific differentiation of tubular cells similarly to its role in fetal epidermal development 6. The continuous expression from fetal kidney through PNL towards papillary RCT suggests that *KRT17* is associated with the development of PNL and subsequently of papillary RCT. This finding indicates a molecular relationship between kidney development and papillary RCT tumorigenesis. The developmental sequences outlined by *KRT17* expression support our hypothesis on the unique natural history of papillary RCT 19.

*KRT17* is a basal/myoepithelial cell keratin the expression of which depends on the position of cells in complex multiplayer human epithelia 25. Expression of *KRT17* has been described in bladder carcinoma, keratoacanthoma and squamous cell carcinoma, oral squamous cell carcinoma, premalignant and malignant squamous lesions of the cervix, all derived from multilayer epithelial cells 7-10. In these cases, the tumorigenesis is similar to that we observed for papillary RCT.

Expression of *KRT17* has also been found in several other types of cancer such as gastric adenocarcinoma, ovarian and breast carcinoma, papillary thyroid carcinoma but not in their corresponding normal tissue 11-16. The neo-expression of *KRT17* in these cases showed a significant correlation with tumor progression and metastasis. We have identified *KRT17* expression in conventional RCCs as an independent negative survival factor indicating a higher risk for postoperative tumour relapse and cancer specific death of patients. Conventional RCC derives from *KRT17* negative proximal tubules of the kidney, which suggests that *KRT17* has not been involved in the development of conventional RCC. Rather, the neo-expression of *KRT17* in conventional RCC can be used as a predictive biomarker similar to gastric, ovarian or breast carcinoma 11-16. Hu and coworkers 16 demonstrated that silencing of *KRT17* in gastric cancer cells inhibited cell proliferation both *in vitro* and *in vivo* conditions, reduced the migration of tumor cells and induced apoptosis by *BCL2* expression. They also showed that silencing *KRT17* leads to cell-cycle arrest at G1/S phase of tumor cells. The clinical, pathological as well as experimental data strongly suggest the involvement of *KRT17* neo-expression in tumor progression.

The key novel findings of this study are, that *KRT17* is expressed in a single-layered epithelia, and that papillary RCT and conventional RCC have distinct natural history. The continuous expression of *KRT17* from fetal kidney tubules towards papillary RCT in adult confirm the relationship between fetal kidney development and tumorigenesis of papillary RCT. And finally, the neo-expression of *KRT17* in aggressive growing conventional RCC is significantly associated with postoperative tumor relapse. The multiple functions of *KRT17* in kidney cancers unequivocally delineates papillary RCTs and conventional RCCs with distinct natural history, which should be taken into account in clinical managements and therapy.

## Figures and Tables

**Figure 1:** Representative pictures of *KRT17* expression in normal kidney, preneoplastic lesions and papillary RCTs. A: Weak *KRT17* positivity at the tip of ureteric bud in connection to the distal part of S-shaped body in foetal kidney. B: Strong *KRT17* staining in each cell of the collecting duct of foetal kidney. C: Selective *KRT17* staining of cells of the medullary collecting in adult kidney. D: *KRT17* positivity in the vast majority of connecting duct cells in adult kidney. E, F: Positive *KRT17* reaction in a tubular and papillary preneoplastic lesion, respectively. G-I: Positive staining with *KRT17* antibody in small, medium size and large cell papillary renal cell tumours, respectively.

**Figure 2:** Expression of *KRT17* in conventional RCC. A: Lack of expression, B: weak cytoplasmic expression, C: strong *KRT17* expression in single tumor cells and D: strong expression in invasive growing tumor cells.

**Figure 3:** Kaplan-Meier estimates of probability for disease-specific survival of patients without metastatic disease at the time of operation. KRT17 negative and positive cases are marked by blue and red curves, respectively.

**Table 1:** Association of KRT17 expression with clinical-pathological parameters of conventional RCCs without metastasis at the time of operation (n=692)

		Nr of cases (692)	KRT17 expression		p-value
			negative	positive	
Gender					0.002
	male	407	338	69	
	female	285	260	25	
Status					<0.001
	AWD	584	528	56	
	DOD	108	70	38	
Size					0.045
	< 4 cm	272	246	26	
	4< x < 7 cm	269	226	43	
	> 7 cm	151	126	25	
T Stadium					0.001
	pT1a	308	275	33	
	pT1b	203	180	23	
	pT2a	78	66	12	
	pT2b	16	14	2	
	pT3a	69	50	19	
	pT3b	15	11	4	
	pT3c	2	2	0	
	pT4	1	0	1	
Grade					<0.001
	G1	458	414	44	
	G2	180	150	30	
	G3	54	34	20	
Stage					<0.001
	I+II	596	527	69	
	III+IV	96	71	25	

AWD - alive without disease; DOD - dead of disease.
